RETRACTED

# Matrine derivate MASM uncovers a novel function for ribosomal protein S5 in osteoclastogenesis and postmenopausal osteoporosis

**DOI:** 10.1038/cddis.2017.394

**Published:** 2017-09-07

**Authors:** Xiao Chen, Xin Zhi, Liehu Cao, Weizong Weng, Panpan Pan, Honggang Hu, Chao Liu, Qingjie Zhao, Qirong Zhou, Jin Cui, Jiacan Su

**Affiliations:** 1 Department of Orthopedics Trauma, Shanghai Changhai Hospital, Second Military Medical University, Yangpu District, Shanghai 200433, China; 2 China-South Korea Bioengineering Center, Jiading District, Shanghai 201802, China; 3 Graduate Management Unit, Shanghai Changhai Hospital, Second Military Medical University, Yangpu District, Shanghai 200433, China; 4 School of Pharmacy, Second Military Medical University, Shanghai 200433, China

## Abstract

Postmenopausal osteoporosis (POMP) is a public health problem characterized by decreased bone density and increased fracture risk. Over-activated osteoclastogenesis plays a vital role in POMP. Here we developed a novel bioactive compound MASM (M19) based on sophocarpine. Although it showed no significant effects on osteogenesis and adipogenesis for bone marrow-derived mesenchymal stem cells (BMSCs) *in vitro*, it could significantly inhibit RANKL/M-CSF induced osteoclastogenesis through suppressing NF-*κ*B, MAPKs and PI3K/Akt pathways *in vitro* and ameliorate bone loss in ovariectomized mice *in vivo*. Ribosomal protein s5 (RPS5) has been identified as a target of M19 and regulates PI3K/Akt, NF-*κ*B and MAPKs pathways in osteoclastogenesis. Overexpressions of RPS5 synergistically inhibited osteoclastogenesis with M19 while silencing RPS5 compromised M19 inhibitory effects on osteoclastogenesis *in vitro*. Among the three pathways, Akt plays a major role in M19 effects. The Akt activator SC_79_ partially reversed the inhibitory effects on osteoclastogenesis by M19 and RPS5-knocking-down. It indicates that RPS5 serves as a potential candidate target for inhibiting osteoclastogenesis and osteoporosis therapy and M19 is a promising agent for POMP treatment.

Osteoporosis is an age-related public health problem characterized by decreased bone density and increased fracture risk.^1^ Primary osteoporosis mainly refers to postmenopausal osteoporosis (POMP) and accounts for a large portion of osteoporosis.^2^ With the population aging, the incidence of primary osteoporosis is dramatically increasing.^3, 4^ Osteoporosis leads to a high incidence of fractures, especially the hip fractures that pose a serious threat to public health.^4^

Osteoporosis is a metabolic bone disease that results from the imbalance between osteoblasts and osteoclasts.^5^ Osteoclasts are derived from the monocyte-macrophage lineage and play a vital role in the pathogenesis of primary osteoporosis, for which inhibiting osteoclast formation and activation remains an important treatment strategy.^6^ As for osteoclastogenesis, receptor activator NF-*κ*B ligand (RANKL)-mediated NF-*κ*B, mitogen-activated protein kinases (MAPKs) and PI3K/Akt pathways are essential, which lead to the activation of nuclear factor of activated T cells (NFATc1) in osteoclast precursors.^7^ RANKL binds to RANK on osteoclast precursors and mature osteoclasts, which activates tumor receptor factor receptor-associated factors 2, 3, 5, 6 (TRAF2, 3, 5, 6), Gab2 and Cbl.^8^ TRAF2 and 6 then activate the TAB1/TAB2/TAK1 complex, which issues an activation of IKK*β* and MAPK, while Gab2 and Cbl bind to RANK-mediated activation of C-Src, PI3 kinase (PI3K) and Akt. Several agents are reported to inhibit OVX-induced osteoclastogenesis through targeting RANKL-induced activations of NF-*κ*B, MAPKs or PI3K/Akt pathways.^9^

RETRACTED

A large body of evidence indicates that the withdrawal of estrogen after menopause is associated with spontaneous increases in pro-inflammatory cytokines and inflammasomes activation, including IL-1, IL-6, and TNF-*α* which contribute to the increased osteoclastogenesis.^10, 11^ Various monomers derived from traditional Chinese herbs showed anti-osteoporosis and osteoclastogenesis inhibitory effects through inhibiting osteoclastogenesis.^12^ Matrine and sophocarpine are the major active components of the Sophora flavescens Ait with various pharmacological effects including anti-fibrosis, anti-tumor, anti-inflammation.^13, 14, 15, 16^ Based on sophocarpine, we synthesized thiosophocarpine and introduced amino groups to the keto beta position to obtain matrine derivatives.^15^ Compared with matrine, the derivative M19 (6aS, 10 S, 11aR, 11bR, 11cS-10-methylamino-dodecahydro-3a, 7a-diazabenzo [de] anthracene-8-thione, C16N3H27S) showed a superior inhibitory effect on NF-*κ*B and Akt pathways.^17^ Our previous study revealed that M19 could inhibit liver fibrosis through inhibiting Akt phosphorylation and ribosomal protein S5 (RPS5) was identified as a direct target to regulate Akt phosphorylation.^16^ RPS5 is an important component of ribosomes and its functions remain largely unknown.^18^ The increasingly accumulated evidence suggests that RPS5 has extraribosomal functions. Since M19 could significantly inhibit NF-*κ*B and Akt pathways, it is highly likely to be able to influence osteoclastogenesis and further OVX-induced bone loss. Our preliminary experiment revealed that matrine could prevent OVX-induced bone loss. To investigate the roles of RPS5 in osteoclastogenesis and the effects of M19 on ovariectomy induced bone loss in mice, we performed this study.

RETRACTED

## Results

### M19 inhibits osteoclastogenesis and osteoclasts function *in vitro*

Before *in vitro* studies, the MTT analysis was performed to determine the appropriate concentration of M19. The results showed that below 11.1 *μ*M, M19 showed no cytotoxic effects (Figure 1b). To investigate the effects of M19 on osteoclastogenesis *in vitro*, we used two standard *in vitro* osteoclast differentiation models, RAW264.7 cells and BMMCs. Without RANKL\M-CSF, no TRAP-positive cells were found on the seventh day. After RANKL induction, the TRAP-positive cells were significantly increased. An addition of M19 in the differentiation cell models significantly reduced the number of TRAP-positive cells in a dose-dependent manner (Figures 1c and d). When incubated with RANKL/M-CSF, RAW264.7 cells differentiated into mature osteoclasts and formed pits on the bone biomimetic synthetic surface. However, the resorbed area was significantly reduced when treated with M19, suggesting that M19 suppressed the functions of osteoclasts (Figure 1e).

### M19 has no effect on M-CSF-induced proliferation and differentiation of BMMs

Osteoclastogenesis process is a multistep process. M-CSF induces bone marrow mononuclear cells (BMMs) to differentiate into pre-osteoclasts which are further induced by RANKL to fuse and form osteoclasts.^19^ To examine which step that M19 taken affects in osteoclastogenesis, we investigated the effects of M19 on BMMs proliferation. Similar to MTT results, M19 had little effect on M-CSF-induced BMMs proliferation at low concentrations (less than 10 *μ*M) (Supplementary Figure S1). Next, we examined the expression levels of RANK and c-Fms by RT-PCR and immunofluorescence to explore the effects of M19 on M-CSF-induced BMMs differentiation. RT-PCR and immunofluorescence assays showed that M19 had little effect on the expression of RANK and c-Fms induced by M-CSF after 12 h (Supplementary Figures S2 and S3). Together, the above results indicated that the inhibitory effects of M19 on osteoclastogenesis were not due to the suppression of M-CSF-induced BMMs proliferation and differentiation into pre-osteoclasts.

### M19 inhibits RANKL-induced osteoclast formation at the early stage, but has little effect on mature osteoclast formation and resorption

To determine the effects of M19 on RANKL-induced pre-osteoclast differentiation into mature osteoclasts, M19 was added to osteoclast differentiation cultures beginning on day 0 to day 5 for BMMs (Figure 2a) and day 0 to day 3 for RAW264.7 cells (Figure 2b). The results indicated that M19 inhibited osteoclastogenesis on the first day and M19 could not inhibit the osteoclastogenesis at later stages. In summary, M19 inhibited RANKL-induced osteoclast differentiation at the early stage.

RETRACTED

### M19 has little effects on osteogenic and adipogenic differentiation of BMSCs

Since M19 affects multiple pathways, whether it affects osteogenesis and adipogenesis of bone marrow mesenchymal cells needs to be answered. To examine whether M19 affects osteogenesis and adipogenesis *in vitro*, we performed the osteogenesis assay and adipogenesist assay. We isolated bone marrow-derived mesenchymal stem cells (BMSCs) from mice, conducted osteogenic and adipogenic induction and added M19 (5 *μ*M). The osteogenic and adipogenic potential of MSCs was assessed 14 days after induction of differentiation by ALP, alizarin red and oil red O staining, respectively. The ALP staining (Supplementary Figure S4) and alizarin red staining (Supplementary Figure S5) showed that M19 had little influence on osteogenesis and adipogenesis of BMSCs. The oil red O staining (Supplementary Figure S6) demonstrated that M19 had little impact on adipogenesis *in vitro*. The results indicated that M19 had little effect on osteogenesis or adipogenesis, which indirectly implied that M19 took effect mainly through affecting osteoclastogenesis.

### M19 inhibits expressions of Osteoclastogenesis-related markers

In RAW264.7 cells, induction with M-CSF and RANKL promoted the expression of osteoclastogenesis-related genes (*P*<0.01) and treatment with M19 significantly inhibited expressions of TRAP, Cathepsin K, TRAF6, MMP-9 and CTR in a dose-dependent manner (*P*<0.05) (Figure 2c).

### M19 combines with RPS5 and suppresses NF-*κ*B, MAPKs and PI3K/Akt pathways in osteoclastogenesis

To determine whether M19 inhibits NF-*κ*B pathway, we performed immunofluorescence staining of P-p65 in the absence and presence of M19 in RAW264.7 cells (Figure 3a). In control group, p65 were located in the cytoplasm, which were unphosphorylated and inactive. After induced with M-CSF and RANKL, most p65 were translocated in the nucleus. The nuclear translocation of p65 was blocked when cells were incubated with 5 *μ*M M19. Ratio of the fluorescence intensity at the nuclear site with whole-cell fluorescence intensity represented the nucleus percentage and it indicated that M-CSF and RANKL induced activation of p65 in RAW264.7 cells (*P*<0.01) and treatment with M19 could inhibit p65 translocation (*P*<0.05) (Figure 3b).

Western blot and semi-quantitative detection showed that induction with M-CSF and RANKL promoted the phosphorylation of p65, p50 and I*κ*Ba (*P*<0.01) in RAW264.7 cells. Treatment with M19 significantly inhibited activation of NF-*κ*B pathway by western blot assays. Meanwhile, we examined the phosphorylation of major subfamilies of MAPKs, P38, JNK, ERK and C-fos and Akt by western blot analysis. The phosphorylated ERK, JNK, C-fos and Akt demonstrated a significant increase after RANKL treatment, and M19 treatment inhibited their phosphorylations (Figure 3c). NFATc1 is a well-known master regulator of osteoclastogenesis and function. To determine whether M19 regulates the expression of NFATc1, we assessed the effects of M19 on NFATc1 mRNA levels. PCR results indicated that expression of NFATc1 was increased after M-CSF and RANKL induction and inhibited after M19 treatment (*P*<0.05) (Figure 3d). All these results indicated that M19 could inhibit NF-*κ*B pathway, MAPK pathway and PI3K/Akt pathway, and reduce the expression of nuclear transcription factor NFATc1.

RETRACTED

A previous study indicated that M19 targeted RPS5. In order to verify the direct combination of M19 and RPS5, we carried out the improved drug affinity responsive target stability (DARTS) experiment. Results showed that, when the PBS treatment group was treated with different concentrations of protease, the protein was degraded more quickly and thoroughly with the increase of the content of protease, but when M19 treatment group was treated with the same group of protease solutions RPS5 degradation was prohibited, which indicated that the protein is not effectively digested by protease and that M19 directly targeted RPS5 (Figure 3e).

### RPS5 regulates osteoclastogenesis

In order to investigate the roles of RPS5 in osteoclastogenesis, the RPS5 gene was silenced and overexpressed in RAW264.7 cells, and the functions of RPS5 in RAW264.7 cells were investigated. After infected with recombinant lentiviral 72 h, the infected efficiency of RAW264.7 cells were close to 100%, demonstrated by the expression of green fluorescence marker GFP. And the expression of RPS5 indicated that RPS5 gene was silenced and overexpressed by virus infection. Significant changes were confirmed in RPS5 overexpressed group and silenced group when compared with the control group (*P*<0.05), and there was no statistical difference between RAW264.7 cell control group and NC control group (*P*>0.05). It indicated that the expression of intracellular RPS5 was not affected by virus infection (Figure 4a). To determine whether inhibition of osteoclastogenesis by M19 was associated with RPS5, the RAW264.7 cell was induced with M-CSF, RANKL and treated with Lv-NC, Lv-shRNA-RPS5 or Lv-RPS5, then incubated with 5 *μ*M M19. Next, the TRAP-positive cells and osteoclast differentiation markers were detected. It indicated that M19 inhibited the osteoclast differentiation and when the RPS5 was silenced, the effects of M19 was compromised and overexpressed the RPS5, further enhancing the function of M19 on osteoclastic differentiation inhibition (Figure 4b).

RETRACTED

The integrity of f-actin ring on the cell membrane is a mark of osteoclastogenesis. Therefore, we carried out f-actin fluorescence on the seventh day of induction. Immunofluorescence assay showed that the expression of f-actin on induction group was continuous and complete. RAW264.7 cells induced with RANKL, treated with 5 *μ*M M19 and infected with Lv-NC group showed that the ring structure of f-actin protein showed obvious fractures and the fluorescence intensity was weakened obviously, indicating that M19 significantly inhibited the osteoclastogenesis and Lv-NC infection had no significant effects on M19 inhibitory effects. The f-actin ring structure of RAW264.7 cells infected with Lv-shRNA-LRPS5 was continuous, and the fluorescence intensity was gradually increased compared with the M19 treatment, which indicated that RPS5 silenced significantly reversed the effects of M19. The f-actin ring structure of RAW264.7 cells infected with Lv-RPS5 was significantly weakened and the ring structure was incomplete, indicating that the high expression of RPS5 enhances the effects of M19 on inhibiting osteoclastogenesis (Figure 4c). Meanwhile, RPS5 silenced could reverse the inhibitory effects of M19 on the expression of TRAP, Cathepsin K, TRAF6, MMP-9 and CTR, and RPS5 overexpressed further enhanced the effects of M19 on the expression of osteoclastogenesis-related markers (Figure 4d).

### RPS5 regulates PI3K/Akt, MAPK and NF-*κ*B pathways

Detection of expression of RPS5 (Figure 5a), P-Akt protein in the above six groups showed that M19 inhibited the Akt phosphorylation and when the RPS5 was silenced, the inhibitory effects of M19 were compromised, and overexpressed RPS5 further enhanced the effects of M19 inhibited PI3K/Akt pathway. It indicated that RPS5 significantly inhibited the activation of the PI3K/Akt pathway (Figure 5b). The phosphorylation of p65, p50 and I*κ*Ba, which was associated with NF-*κ*B pathways, was also inhibited by M19. RPS5 promoted or suppressed the effects of M19 (Figure 5c). The phosphorylation of ERK, JNK, associated with MAPK pathway, and phosphorylation of C-fos, an important downstream transcription factor of MAPK pathway indicated that RPS5 also affected the MAPK pathway (Figure 5d).

### Akt agonist reverses M19 effects on osteoclastogenesis

We examined the effects of Akt agonists on osteoclastogenesis. BMMs and RAW264.7 cells were induced with M-CSF, RANKL and treated with M19 or SC_79_ (5 *μ*g/ml), an Akt agonist. When RPS5 was overexpressed, the osteoclastogenesis was inhibited as shown in group 4 in Figures 4 and 5. We added AKT agonist SC_79_ (5 *μ*g/ml) into the RPS5 overexpressed cells which were then induced with M-CSF and RANKL. TRAP results showed that SC_79_ did reverse the inhibitory effects of RPS5 on osteoclastogenesis (Figure 6a). In BMMs cells, TRAP staining results showed that the Akt agonist could reverse the effects of M19 on osteoclastogenesis (Figure 6b). In RAW264.7 cells, M-CSF and RANKL promoted the expression of osteoclastogenesis-related genes and treatment with M19 significantly inhibited expression of TRAP, Cathepsin K, TRAF6, MMP-9 and CTR. SC_79_ reversed the effects of M19 on osteoclastogenesis (Figure 6c). It suggested that RPS5 probably mainly take effects through the PI3K/Akt pathway.

RETRACTED

### M19 inhibits ovariectomy-induced bone loss *in vivo*

To examine whether M19 prevented OVX-induced bone loss, we used the OVX mouse model to mimic menopause-induced bone loss in women. hematoxylin and eosin (H&E) staining showed that, after 6 weeks, OVX mice exhibited a significant loss of trabecular bone when compared with the sham-operated mice. M19 significantly prevented the OVX-induced bone loss. (Figure 7a). The TRAP staining indicated that the osteoclastogenesis was increased in OVX group and M19 administration significantly reduced the number of osteoclasts (Figure 7b). These results were further corroborated by Micro CT. The two-dimensional structure and three-dimensional structure were showed in the figure and as measured by BV/TV, BS/TV, Tb.pf, Tb.N and bone mineral density (BMD) (Figures 7c and d).

We next examined whether M19 prevented OVX-induced bone loss by inhibiting osteoclast activity. Compared with OVX mice, OVX mice treated with M19 displayed a decreased serum IL-6, TNF-*α* and TRAcp5B level (*P*<0.05), which reflected the osteoclast activity *in vivo* (Figure 7e). The results of bone marrow ELISA are consistent with the serum results (Supplementary Figure S7). Because bone remodeling is regulated by bone resorption and bone regeneration, we also investigated the effects of M19 on osteoblasts, the serum osteocalcin (Figure 7e), a serologic marker of osteoblast function. No significant difference was found between OVX group and treatment group. The results above indicated that M19 inhibited osteoclastogenesis in OVX mice *in vivo* and prevented the OVX-induced bone loss.

## Discussion

In this study, we found that M19 significantly ameliorated bone loss in ovariectomized mice *in vivo*. *In vitro* we demonstrated that M19 could inhibit RANKL/M-CSF-induced osteoclastogenesis during which RPS5 was significantly downregulated, but was stablized by M19. DARTS test confirmed that M19 targeted RPS5. Overexpressions of RPS5 compromised activation of NF-*κ*B, MAPKs and PI3K/Akt pathway and inhibited osteoclastogenesis synergistically with M19. Silencing RPS5 could reduce the inhibitory effects of M19. Akt activator could reverse the M19 effects. The results indicated that RPS5 could serve as a potential target for inhibiting osteoclastogenesis-related diseases. It probably affected the activation of the NF-*κ*B, MAPKs and PI3K/Akt pathway, in which PI3K/Akt played a major role as previously reported^16^ (Figure 8).

RETRACTED

Bone regeneration and resorption balance is delicately regulated by osteoblasts and osteoclasts.^20^ In osteoporosis, the balance is disrupted with increased osteoclastogenesis and decreased osteogenesis due to various causes like estrogen deficiency, aging, inflammation, which results in net bone loss.^21, 22, 23^ Excessive bone resorption by over-activated osteoclasts plays a vital role in the pathogenesis of osteoporosis. Inflammation plays an important role in the pathogenesis of POMP.^24, 25^ In ovariectomized mice, serum levels of pro-inflammatory cytokines such as TNF-*α*, IL-1*β* were significantly upregulated. On one hand, increased pro-inflammatory cytokines over-activates osteoclastogenesis which accelerates bone resorption.^26, 27^ On the other hand, aggravated inflammation increases oxidative stress and inhibits osteogenesis.^28, 29^ Wnt4 could prevent skeletal aging and inflammation by inhibiting NF-*κ*B and ameliorates inflammation.^17, 30^ Thus, inhibiting osteoclastogenesis through anti-inflammation becomes an important strategy in osteoporosis treatment and screening the potential osteoclastogenesis inhibitor is a promising strategy for new anti-osteoporosis drug development.

Traditional Chinese herbs provide abundant resources for novel therapeutic agents for osteoporosis.^31^ Matrine, oxymatrine and derivatives have exhibited various pharmaceutical effects, including inhibition of inflammation,^15^ liver fibrosis^16^ and tumor growth.^32^ Based on matrine, we synthesized M19 that exhibited better anti-inflammatory effects than matrine.^15, 16^ In this study, we found that serum levels of TRAcp5B, TNF-*α* and IL-6 were significantly elevated in ovariectomized mice and decreased by M19 treatment. *In vivo*, M19 significantly reduced bone loss in ovariectomized mice and inhibited osteoclastogensis testified by the decreased serum TRAcp5B level and TRAP staining.

Before *in vitro* studies, we first performed MTT analysis. The results showed that below 11.1 *μ*M, M19 had no cytotoxic effects. Thus, we selected 1, 2 and 5 *μ*M for *in vitro* studies to rule out the cytotoxic effects of M19. M-CSF and RANKL are essential for osteoclast differentiation, in which M-CSF induces osteoclast precursor cells proliferation and differentiation while RANKL induces subsequent differentiation.^7, 33^ After RANKL binding to RANK on the surface of osteoclast precursor cells, TRAFs were recruited and MAPKs p38, JNK and canonical NF-*κ*B pathways were activated.^34, 35^ Besides, Akt/PKB could be activated through interactions between TRAF6 and Cbl scaffolding proteins.^36, 37^ In this study, we found that M19 could suppress M-CSF and RANKL-induced osteoclastogenesis demonstrated by TRAP staining in both BMMCs and RAW264.7 cells and inhibit PI3K/Akt, NF-*κ*B and MAPKs pathways as well as the expression of NFATc1, the most important osteoclastogenesis-related transcription factor.^38, 39, 40^

RETRACTED

A previous study demonstrated that M19 inhibited hepatic stellate cells (HSC) activation and protected liver fibrosis through stabilizing RPS5 in HSC. After RPS5 was downregulated through RNA interference, liver fibrosis was aggravated.^16^ It indicates that RPS5 is an important upstream regulator of Akt pathway.^16^ The increasingly accumulated evidence suggests that RPS5 has extraribosomal functions. It is reported that RPS5 could interact with hepatitis C virus and cricket paralysis virus.^41, 42^ Casein kinase II could phosphorylate RPS5, which plays an important role in protein trafficking from cytoplasm to nucleoli.^43^ In this study, we first confirmed the combination of M19 and RPS5 by a DARTS test in RAW264.7 cells. Since M19 displayed a significant inhibitory effect on osteoclastogenesis, probably RPS5 has a role in osteoclastogenesis. Previous studies only explored the roles of RPS5 in Akt phosphorylation,^16^ the effects of RPS5 on cell signalling remain largely unkown. Thus, in this study we explored the roles of RPS5 in osteoclastogenesis as well as in PI3K/Akt, NF-*κ*B and MAPKs pathways.

Osteoclastogenesis significantly decreased RPS5 level while M19 stablized RPS5. After RPS5 was silenced, the osteoclastogenesis inhibitory effects of M19 were drastically compromised as demonstrated by the increased number of TRAP-positive cells and elevated expressions of osteoclastogenesis-related markers. When it was overexpressed, the osteoclastogenesis inhibitory effects of M19 were enhanced when compared with single M19 administration.

RANKL/M-CSF treatment significantly induced phosphorylations of Akt, p65, p50, I*κ*Ba, ERK and JNK, which were inhibited by M19. Although p-p38 was also increased, the difference was not statistically different. Akt, p65, p50, I*κ*Ba, ERK and JNK phosphorylations were reduced accompanied with RPS5 overexpression and increased with RPS5 silencing. All these results demonstrated that RPS5, stabilized by M19, regulated osteoclastogenesis through the PI3K/Akt, NF-*κ*B and MAPKs pathways.

RETRACTED

It is reported that Akt simply could influence osteoclastogenesis.^44^ To further investigate the relationships of RPS5 and Akt in osteoclastogenesis, we used SC_79_ as an Akt activator.^45^ The osteoclastogenesis inhibitory effects of M19 were significantly compromised demonstrated by increased expressions of osteoclastogenesis-related markers. It implied that M19 inhibited the osteoclatogenesis mainly through the Akt pathway.

In this study, we used Trap, Cathepsin K, TRAF6 CTR and MMP-9 as osteoclastogenesis-related markers based on previous reports.^46, 47^ Matrix metalloproteinases (MMPs), also known as matrixins, are calcium-dependent zinc-containing endopeptidases.^48^ The MMPs belong to a larger family of proteases known as the metzincin superfamily.^49^ Collectively, these enzymes are capable of degrading all kinds of extracellular matrix proteins, but also can process a number of bioactive molecules. MMP-9 is implicated in osteoclast-induced bone resorption.^50, 51^ Increased expression of MMP-9 has been described in RA patient serum.^52^ The previous study suggested that MMP-9 was an important downstream effector molecule driving pathologic systemic bone loss observed in osteoporosis.^53^ Many studies employed MMP-9 as osteoclastogenesis-related markers.^12, 47, 54^ Our study demonstrated that M19 inhibited expressions of MMP-9 during osteoclastogenesis.

Our study for the first time demonstrates RPS5 affected multiple cell signaling pathways in which Akt plays a major role and indicates that RPS5 is an important up-stream regulator and a promising candidate target for primary osteoporosis treatment. It is possible that the roles of RPS5 have been underestimated currently and remain largely unknown. It is not only a vital structure for ribosomes, but also contributes to important intracellular cell signaling transduction. However, the exact mechanism of RPS5 affecting NF-*κ*B, MAPK and Akt pathways is far more complicated than what we deduce. ChIP analysis could help to reveal the relationship of RPS5 with DNA and IP assay could clarify protein–protein interactions. Nevertheless, currently there has been no evidence that RPS5 could directly affect DNA transcription and three pathways (NF-*κ*B, MAPK and Akt) involve tens of proteins required to be testified sequentially. To clarify the exact RPS5–DNA and RPS5–Protein relationships in this study is quite challenging, however remain very intriguing.

Some questions still require to be answered. After RPS5 was silenced, the inhibitory effect of M19 was compromised; however they still existed when compared with induction. Possibilities are that RPS5 was knocked-down instead of being completely knocked-out and M19 acted through interacting with other targets and pathways although mainly through RPS5/Akt. How RPS5 interacts with Akt, whether M19 has novel targets in osteoclastogenesis and how RPS5 affects primary osteoporosis *in vivo* require to be solved before it is clinically applied.

RETRACTED

## Materials and methods

### Regents

13-methylamino-18-thiomatrine (M19, Figure 1a) was supplied by Prof. Hu, HG from the School of Pharmacy, Second Military Medical University. Briefly, sophocarpine was transformed into thiosophocarpine in high yield by treatment with Lawesson’s reagent. Then, M19 was synthesized by reaction of thiosophocarpine with NH_2_CH_3_. SC_79_ purchased from Abcam (Cambridge, MA, USA). M19 was made into maleate and dissolved in normal saline as vehicle for use.

### MTT assay

The MTT assay was performed according to the manufacturer’s instructions. The concentration of MTT solution was 5 mg/ml. BMM cells were cultured at a density of 100 *μ*l (10 × 10^4^/ml) per well on a 96-well plate for 24 h incubation. Cells were then cultured with various concentrations of M19 (1.2, 3.7, 11.1, 33.3 and 100 *μ*M) for 48 h. The MTT solution was added at 10 *μ*l per well and incubated for 2 h. Absorbance was measured at 490 nm using ELISA plate reader.

### Osteoclastogenesis assay *in vitro*

To evaluate the effects of M19 on osteoclastogenesis *in vitro*, BMMs were isolated from the femur bone marrow of C57BL/6 mice at 6 weeks of age as previously reported.^55^ BMMs were cultured under the 37 °C and 5% CO_2_ condition. Cells of the third generation were collected and induced with M-CSF (20 ng/ml) and RANKL (50 ng/ml) in the absence or presence of various concentrations of M19 (1, 2, 5 *μ*mol/l). At the seventh day after staining with tartrate-resistant acid phosphatase (TRAP) (Sigma-Aldrich, St. Louis, MO, USA) according to the manufacturer’s protocol. TRAP^+^ cells with more than three nuclei were counted as osteoclasts. For RAW264.7 cells (offered by Prof. Hou Jin from the department of immunology of the second military medical university), protocols were similar to the mentioned above.

To determine the effects of RPS5 on the inhibition of osteoclastogenesis by M19, RPS5 was overexpressed or silenced in RAW264.7 cells by lentivirus infection. The RAW264.7 cells were induced to osteoclasts and treated with M19. After 7 days, the osteoclasts were stained by TRAP and TRAP^+^ cells were counted. All the experiments were carried out three times.

### Pit formation assay

To further examine the effects of M19 on osteoclast function, we examined how M19 affected RANKL-induced osteoclast pit formation on bone biomimetic synthetic surface, which represent the function of mature osteoclasts. RAW264.7 cells were seeded (3 × 10^3^ cells/well) on bone biomimetic synthetic surface-coated plates (Corning, St. Lowell, MA, USA) in the absence or presence of 100 ng/ml RANKL with or without M19 of various concentrations. After 7 days, the osteoclast resorbing pits at the bone biomimetic synthetic surface were observed using a light microscope (OLYMPUS-BX53). Pit areas were quantified using Image-Pro Plus software.

RETRACTED

### Immunofluorescence staining

To determine the effects of M19 on the nuclear translocation of p65, the RAW264.7 cells after induction with RANKL and M-CSF in the absence and presence of M19 (5 *μ*mol/l) were examined by immunofluorescence as previously reported.^56^ RAW264.7 cells of each group were fixed with 4% PFA for 15 min and washed with 0.2% Triton X-100 in PBS for 10 min. Then clogged with 1% BSA in PBS and treated with anti-p65 antibody (Abcam), followed by biotinylated goat anti-mouse IgG antibody (Abcam) and fluorescein-conjugated streptavidin. The cells were counterstained with propidium iodide. Three fields of vision were randomly selected and counted 10 cells per field.

### Drug affinity responsive target stability test

To confirm that M19 targets RPS5, we carried out a DARTS test.^57^ Ten micrograms of mouse recombinant protein RPS5 (marked by His) was dissolved in 1 ml of sterile water, and 10 *μ*l of halt protease and phosphatase inhibitor cocktail was added and placed on ice. Three hundred microliters of the above protein solution was divided into two centrifuge tubes, and placed at 25 °C for 10 min. M19 (100 *μ*M) was added into a centrifuge tubes at 25 °C for 30 min and PBS was added into the other centrifuge tubes. The ratio of RPS5 and protease (10 mg/ml) were 1:0, 1:64 and 1:32, and was incubated at 25 °C for 30 min. The concentration of His was detected by western blot. The concentration of the separated gel of western blotting was 10% and anti-His was diluted 1:1200.

### Preparation of lentivirus and lentivirus infection of RAW264.7 cells

#### Construction of pSIH1-shRNA-RPS5 and pCDH-RPS5 plasmid

A siRNA sequence complementarily binding to mouse RPS5 was chosen. The target sequences of siRNA (5′-GCTCATGACTGTGCGAATT-3′) are homologous to RPS5 (NM_009095.2), respectively. The oligonucleotide templates of these shRNAs were chemically synthesized and cloned into the linear pSIH-H1-copGFP shRNA Vector (System Biosciences, Palo Alto, CA, USA) that was obtained through digestion by *Bam*HI and *Eco*RI and purification by agarose gel electrophoresis. An invalid siRNA sequence (5′-GAAGCCAGATCCAGCTTCC-3′) was used as a negative control (NC). Sequencing was used to confirm the vectors constructed (pSIH-shRNA-RPS5 and pSIH-NC).

RETRACTED

Total mouse RNA was extracted by using trizol (Invitrogen, Carlsbad, CA, USA) and reversely transcribed into cDNA, which was used for PCR amplification of RPS5 gene using the primers as following: RPS5-forward primer: 5′-GCTCTAGA (*Xba*I) GCCACC (kozak) ATGACTGAGTGGGAAGCA-3′ RPS5-reverse primer: 5′-CGGGATCC (*Bam*HI) TCAGCGGTTAGACTTGG-3′. The product was cloned to pcDH-GFP Lentivector (CD511A-1, System Biosciences) to construct the RPS5 expression vector pcDH-RPS5.

The endotoxin-free plasmids of the recombinant vectors (pSIH-NC, pSIH-shRNA-RPS5 and pcDH-RPS5) were prepared after being verified by sequencing and co-transfected with pPACK Packaging Plasmid Mix (System Biosciences) into 293 T cells line to produce the lentiviruses of Lv-shRNA-RPS5, Lv-NC and Lv-RPS5. The packaging and titer measurement were performed completely in accordance with the instruction of kit.

#### Packaging and production of recombinant lentivirus

One day before transfection, 293TN cells were seeded into 10 cm dishes. Two micrograms of each pSIH1-shRNA-RPS5 vector or pSIH-NC or pSIH-shRNA-RPS5 and 10 *μ*g pPACK Packaging Plasmid Mix (System Biosciences) were co-transfected using Lipofectamine 2000 (Invitrogen) in accordance with the manufacturer’s protocol. The medium was replaced with DMEM plus 1% FBS. Forty-eight hours later, the supernatant was collected and then cleared by centrifugation at 5000 × *g* at 4 °C for 5 min, and passed through a 0.45 *μ*M PVDF membrane (Millipore, Shanghai, China). The titer of virus was determined by gradient dilution. The packaged lentiviruses were named as Lv-shRNA-RPS5, Lv-NC and Lv-RPS5.

#### Lentivirus infection of RAW264.7 cells

RAW264.7 cultures were made into cell suspension by trypsinization, which was seeded on six-well plates and cultured under the same conditions as before. The cells were divided into four groups: control group (not infected); cells infected with Lv-NC; cells infected with Lv-shRNA-RPS5; and cells infected with Lv-RPS5. After cultured overnight, the cells were added with corresponding lentiviral solution at MOI=20, and cultured for 72 h. Then the cells were collected and subjected to RPS5 measurement by western blotting for determining the genetic intervention efficiency.

### Western blot

To determine the effects of M19 on expressions of osteoclastogenesis-related markers, the total cellular proteins of each group RAW264.7 cells were extracted and TRAP, Cathepsin K, TRAF6, MMP-9 and CTR were detected by western blot. To evaluate the effects of M19 on NF-*κ*B pathway, MAPK pathway, PI3K/Akt pathway and RPS5 expressions levels, the phosphorylation of P50, P65 and I*κ*Ba protein; phosphorylation of ERK, JNK, C-fos and P38 protein; phosphorylation of AKT and expression of RPS5 was determined by western blot.

RETRACTED

To investigate the roles of RPS5 on the osteoclastogenesis, we detected the TRAP, Cathepsin K, TRAF6, MMP-9, CTR protein and the phosphorylation of P50, P65, I*κ*Ba, ERK, JNK, C-fos, P38 and AKT protein from the RAW264.7 cells on the third day after induction, in which RPS5 was overexpressed or silenced.

The total protein was extracted from the cells using M-PER mammalian protein extraction reagent (Pierce, Rockford, IL, USA). Equal amounts of protein (10 *μ*g per lane) estimated by a bicinchoninic acid (BCA) protein assay kit (Pierce) were loaded onto (11%) SDS-PAGE gels and transferred onto nitrocellulose membranes. The blots were probed with a monoclonal antibody against human anti-TRAP (1:350), anti-Cathepsin K (1:500), anti-TRAF6 (1:250), anti-MMP-9 (1:400), anti-CTR (1:200), anti-p65 (1:350), anti-P-p65 (1:500), anti-p50 (1:250), anti-P-p50 (1:400), anti-I*κ*Ba (1:350), anti-P-I*κ*Ba (1:500), anti-ERK (1:200), anti-P-ERK (1:400), anti-JNK (1:500), anti-P-JNK (1:400), anti-p38 (1:300), anti-P-p38 (1:300), anti-RPS5 (1:150), anti-AKT1 (1:250), anti-P-AKT1 (1:400), anti-C-fos(1:600), anti-P-C-fos (1:400) and anti-beta actin (1:1000) (Santa Cruz, Dallas, TX, USA), followed by the secondary HRP-conjugated anti-mouse/rabbit antibody (Santa Cruz). After washing, the bands were detected by chemiluminescence and imaged with X-ray films. Beta actin was used as an endogenous reference for normalization.

### F-actin ring formation assay

RAW264.7 cells were seeded onto six-well culture plates (2 × 10^6^ cells/well) and cultured for 24 h. RAW264.7 cells were fixed with 4% PFA in PBS for 10 min. The cells were permeabilized with 0.1% Triton-X 100 in PBS for 5 min and incubated with rhodamine-conjugated phalloidin (Biotium, Fremont, CA, USA) to visualize F-actin. All the experiments were carried out three times. Anti-F-actin that marked with FITC was purchased from Abcam and diluted to 1:600.

### PCR analysis

Total RNA was prepared from cells using Trizol reagent. The forward and reverse primers of NFATc1 (NM_016791.4) were 5′-ATCGCCCAGGCACTCCCCATCCAG-3′, 5′-GCTGCCGGCCATTGAGACTGTA-3′. The primer sequence of *β*-actin was 5′-GCAAT GCCTG GGTAC ATGGT GG-3′. Complementary DNA synthesis and quantitative analysis were performed with Super Script Reverse Transcriptase (Invitrogen) according to the manufacturer’s protocol. Amplification was performed using ABI ViiA7 Real Time System (Applied Biosystems, Foster City, CA, USA) by means of incorporation of SybrGreen fluorescent dye as reported. Beta actin was used as a reference to normalize the NFATc1 level using the 2_ΔΔ_Ct method.

RETRACTED

### Animals and experimental design

All experiments were implemented in the specific pathogen free animal laboratory of Changhai hospital (Shanghai, China). Female 6-week-old C57 mice were purchased from Slack (Shanghai, China). Maintenance, use and treatment of all animals in this experiment were in accordance with accepted standards of the Ethics Committee of SMMU. The sample size calculation was based on our preliminary experiments with 90% power, 5% risk of type I error and 10% risk of type II error. The mice were divided into three groups with six mice in each: sham group: mice receiving sham operation; ovariectomy (OVX) group: mice treated with vehicle; and treatment group: OVX mice treated with M19. The mice in OVX and treatment group were injected intraperitoneally (i.p.) with vehicle and M19 (200 mg/kg) every day. After 6 weeks, all mice were anesthetized with chloral hydrate. Then, the femur and arterial blood were collected. Blood was centrifuged with 3000 r.p.m., 5 min and supernatant was conserved at −80 °C. No significant adverse effects were observed in treatment group.

### Histologic analysis

Femur samples were fixed by 4% paraformaldehyde for 4 days. Then, they were decalcified for 2 weeks by 10% tetracycline-EDTA. Paraffin-embedded sections (4 *μ*m) from each distal femur metaphysis were prepared with H&E staining and TRAP staining for histologic observation. Histologic measurements and images were obtained under a microscope with × 40 magnification (OLYMPUS-BX53). Trabecular bone area within the selected area was calculated and the number of osteoclasts in the region was counted by TRAP staining by Image-Pro Plus software.

### Bone structure analysis

The femur bone structure was analyzed using micro-computed tomography (Micro CT) (Skyscan1172, Antwerp, Belgium). The analysis conditions were 80 kv, 124 *μ*A and resolution was 8 *μ*m. Under this condition, 100 section planes were analyzed from the growth plate. Structural parameters for metaphyseal region and trabecular bone were analyzed using the built-in software. BMD was measured, and the trabecular parameters were evaluated as the bone volume/total volume (BV/TV), trabecular number (Tb. N) and trabecular pattern factor (Tb. Pf) and bone surface area was expressed per unit total volume (BS/TV). Two-dimensional and three-dimensional bone structure image slices were reconstructed.

### Serum biochemistry

Blood was collected from the left ventricle and bone marrow was collected from the femur. Serum levels of IL-6, TNF-*α*, TRAcp5B and OCN were measured by IL-6, TNF-*α*, TRAcp5B and OCN ELISA kits (Anogen, Canada) according to the manufacturer’s instructions.

RETRACTED

### Statistical analysis

Data were expressed as means±S.D. The two independent-sample *t*-test was used for comparisons between two groups. In cases of comparison involving more than two groups, a one-way ANOVA was used. Statistical significance was considered as *P*<0.05.

## Publisher’s Note

Springer Nature remains neutral with regard to jurisdictional claims in published maps and institutional affiliations.

## Figures and Tables

**Figure 1:** M19 inhibits osteoclastogenesis *in vitro*. All the experiments were carried out three times and the average was taken. (**a**) Chemical structure of M19 and the synthesis process. (**b**) MTT analysis of M19 cytotoxic effects in RAW264.7 cells. (**c**) Formation of TRAP-positive cells from BMMCs and quantification of osteoclast. (**d**) Formation of TRAP-positive cells from RAW264.7 cells and quantification of osteoclast. (**e**) The resorption area on the bone biomimetic synthetic surface was quantified by image analysis (*P<0.05, **P<0.01, ***P<0.001)

**Figure 2:** M19 inhibits osteoclastogenesis at early stage and inhibits expressions of osteoclastogenesis-related markers. (**a**) Effect of M19 on RANKL-induced primary osteoclast precursor differentiation at different stage. (**b**) Effect of M19 on RANKL-induced RAW264.7 cell differentiation at different stages. (**c**) Western blot and optical density analysis of expression of Trap, Cathepsin K, TRAF 6, MMP9 and CTR with Beta actin as reference. ①RAW264.7 cells; ② RAW264.7 cells induced with M-CSF, RANKL and PBS; ③ RAW264.7 cells induced with M-CSF, RANKL and treated with 1 *μ*M M19; ④ RAW264.7 cells induced with M-CSF, RANKL and treated with 2 *μ*M M19; ⑤RAW264.7 cells induced with M-CSF, RANKL and treated with 5 *μ*M M19 (*P<0.05, **P<0.01 *versus* ②)

**Figure 3:** M19 Suppresses NF-*κ*B, MAPKs and PI3K/Akt pathways in osteoclastogenesis and targets RPS5. (**a**) M19 inhibits RANKL-induced p65 nuclear translocation. RAW 264.7 cells were pretreated with or without M19 (5 *μ*M) and then stimulated with or without 50 ng/ml of RANKL for 20 min. The localization of p65 was visualized by immunofluorescence analysis. (**b**) Ratio of the fluorescence intensity at the nuclear site with whole cell fluorescence intensity. (**c**) Phosphorylation of p65, p50, I*κ*Ba, EPK, JNK, p38, Akt and c-fos protein, which was associated with NF-*κ*B, MAPK and PI3K/Akt pathway. (**d**) Semi-quantitative detection of NFATc1 gene expression in three groups. (**e**) Content of RPS5 in each group and detection of RPS5 protein content after enzymatic hydrolysis. ①Control; ② RANKL/M-CSF induction and treated with PBS; ③ RANKL/M-CSF induction and treated with 5 *μ*M M19

**Figure 4:** RPS5 regulates osteoclastogenesis. (**A**) Left: fluorescence of cells infected with lentivirus after 72 h. (**a** and **b**) was infected with Lv-RPS5 and (**c** and **d**) was infected with Lv-shRNA-RPS5. Right: Detection of intracellular RPS5 protein expression, MOI=20. (**B**) Formation of TRAP-positive cells from RAW264.7 cells in the six groups. (**C**) Actin ring structures of osteoclasts in the six groups. (**D**) TRAP, Cathepsin, TRAF6, MMP9 and CTR were detected in different treatment groups. ①RAW264.7 cells; ② RAW264.7 cells induced with M-CSF, RANKL and PBS; ③ RAW264.7 cells infected with Lv-NC, induced with M-CSF, RANKL and treated with 5 *μ*M M19; ④ RAW264.7 cells infected with Lv-RPS5; ⑤ RAW264.7 cells infected with Lv-shRNA-RPS5, induced with M-CSF, RANKL and treated with 5 *μ*M M19. ⑥ RAW264.7 cells infected with Lv-RPS5, induced with M-CSF, RANKL and treated with 5 *μ*M M19 (**P<0.01, *P<0.05 *versus* ②)

**Figure 5:** RPS5 regulates PI3K/Akt, MAPKs, NF-*κ*B pathway. (**a**) Changes of RPS5 during osteoclastogenesis. (**b**) Phosphorylation of Akt. (**c**) Phosphorylation of p65, p50 and I*κ*Ba. (**d**) Phosphorylation of ERK, JNK, p38 and c-fos. ①RAW264.7 cells; ② RAW264.7 cells induced with M-CSF, RANKL and PBS; ③ RAW264.7 cells infected with Lv-NC and induced with M-CSF, RANKL and treated with 5 *μ*M M19; ④ RAW264.7 cells infected with Lv-RPS5; ⑤ RAW264.7 cells infected with Lv-shRNA-RPS5 and induced with M-CSF, RANKL and treated with 5 *μ*M 19; ⑥ RAW264.7 cells infected with Lv-RPS5 and induced with M-CSF, RANKL and treated with 5 *μ*M M19

**Figure 6:** Akt agonist reverses the M19 effects. (**a**) AKT agonist reverses RPS5-induced osteoclast inhibition. (**b**) Formation of TRAP-positive cells from BMMCs and treated with M19 or Akt agonist. (**c**) Western blot of Trap, Cathepsin K, TRAF6, MMP9 and CTR. ①RAW264.7 cell; ② RAW264.7 cells induced with M-CSF and RANKL; ③ RAW264.7 cells induced with M-CSF, RANKL and treated with PBS; ④ RAW264.7 cells induced with M-CSF, RANKL and treated with 5 *μ*M M19; ⑤ RAW264.7 cells induced with M-CSF, RANKL and treated with 5 *μ*M M19 and SC_79_ (**P<0.01, *P<0.05 *versus* ②)

**Figure 7:** M19 reduces ovariectomy-induced bone loss *in vivo*. (**a**) Representative H&E staining of distal femoral sections and quantification of trabecular area from each group 6 weeks after the operation. (**b**) Representative TRAP-stained histologic distal femur sections from sham, OVX and OVX+M19 group. (**c**) Micro CT analysis of the distal femur from sham, OVX and OVX+M19 group. (**d**) Calculations of trabecular number (Tb.N), bone surface area/total value (BS/TV), bone value/total value (BV/TV), bone mineral density (BMD) and trabecular pattern factor (Tb.Pf). (**e**) Serum IL-6, TNF-*α*, TRAcp 5B and OCN were examined (*P<0.05, **P<0.01, ***P<0.001)

**Figure 8:** A schematic diagram of the mechanism by which M19 inhibits osteoclast differentiation. RANKL-RANK signaling induces NFATc1 expression through NF-*κ*B, MAPKs and PI3K/Akt pathways. M19 acts on the RPS5 and blocks NF-*κ*B, MAPKs and PI3K/Akt pathways and, subsequently, suppresses NFATc1 expression
